# Correlation between Serum Oxidative Stress Level and Serum Uric Acid and Prognosis in Patients with Hepatitis B-Related Liver Cancer before Operation

**DOI:** 10.1155/2022/1964866

**Published:** 2022-04-11

**Authors:** Maowen Yu, Chaozhu Zhang, Hongbo Tang, Chaohui Xiao

**Affiliations:** ^1^Department of Clinical Lab, Jintang Hospital, West China Hospital, Sichuan University Jintang First People's Hospital, Chengdu 610400, China; ^2^Gastroenterology Department, Chinese PLA Army 951 Hospital, Kuerle 841000, China; ^3^Department of Hepatobiliary Surgery, Fifth Medical Centre of Chinese PLA General Hospital, Beijing 100039, China

## Abstract

Aiming to explore the correlation between preoperative serum oxidative stress level and serum uric acid and prognosis of hepatitis B-related liver cancer, the clinical data of 712 patients with hepatitis B-related liver cancer from January 2019 to December 2020 were retrospectively analyzed. By using the receiver operating curve, the optimal critical values of preoperative superoxide dismutase (SOD), malondialdehyde (MDA), and serum uric acid (SUA) are determined. The single-factor and multifactor Cox models are applied to screen out the suspicious factors affecting the prognosis of patients with hepatitis B-related liver cancer. According to the survival status of patients, the optimal thresholds of SOD, MDA, and SUA before operation were 58.055/mL, 10.825 nmol/L, and 312.77 nmol/L, respectively. The results of univariate analysis show that the prognosis of patients is significantly correlated with preoperative SOD, MDA, and SUA levels and TNM staging (*P* < 0.05). Additionally, multivariate analysis demonstrates that preoperative SOD < 58.055 U/mL and SUA ≥ 312.770 mmol/L and TNM stage III-IV are independent risk factors for postoperative prognosis (*P* < 0.05). Our study suggests that SOD, SUA, and TNM staging have certain value in judging the early prognosis of patients with hepatitis B-related liver cancer. Patients with high preoperative SOD level and low preoperative SUA level can obtain better prognosis.

## 1. Introduction

Hepatocellular carcinoma (HCC) is one of the common malignant tumors in the Chinese population. According to the 2014 World Health Organization report, the number of new cases and deaths of HCC in China is huge, and it has been ranked first in the world for many years. China has a large population and a high rate of HBV infection, leading to about half of the new cases of liver cancer each year [1]. At present, the staging system of hepatocellular carcinoma (HCC) is not ideal for predicting the prognosis of patients with liver cancer after surgical resection, and the recurrence rate after 5 years is more than 50% [2]. An epidemiological survey showed that patients with hepatitis B-related liver cancer had a lower 5-year survival rate of only 20%, with poor prognosis and a serious threat to their lives and health [3]. Therefore, early detection and identification of these patients with postoperative recurrence and targeted intervention are essential. In recent years, the role of oxidative stress in tumors has gradually attracted attention.

Studies have shown that patients with cancer have detected an increase in oxidative stress level before treatment, and it is also related to postoperative prognosis, which is conducive to the development of appropriate individualized treatment for patients [4]. In addition, serum uric acid is another important indicator to evaluate the prognosis of cancer. Related studies have confirmed that elevated serum uric acid levels are associated with the incidence and mortality risk of various diseases such as gastric cancer, colon cancer, renal cell carcinoma, and liver cancer [5]. Clinical studies have confirmed that hyperuricemia not only causes gout but also is closely related to kidney disease, cardiovascular disease, and endocrine and metabolic diseases. Hyperuricemia is an important and independent risk factor for cardiovascular disease and cardiovascular risk factors, such as hypertension, hyperlipidemia, type 2 diabetes, obesity, insulin resistance, and metabolic syndrome [6]. Many studies have shown that the increase of SUA level is an independent risk factor for malignant tumor occurrence and poor prognosis [7, 8]. The proinflammatory properties of SUA may play an important role in the occurrence and development of cancer [9].

Therefore, the analysis of serum oxidative stress and uric acid levels in patients with hepatitis B-related lung cancer is of great significance to understand the occurrence and development of the disease. In this study, the serum oxidative stress and uric acid levels in patients with hepatitis B-related lung cancer before operation were detected to analyze the relationship between the two and the prognosis and survival of patients after operation, so as to use them as effective indicators for prognosis judgment in clinical practice.

## 2. Related Work

Existing works demonstrate that the infection of hepatitis B virus (HBV) in patients with chronic infection is an important reason for the transformation of liver cirrhosis into hepatocellular carcinoma. China is a big country with hepatitis B, in which 60% to 80% of liver cirrhosis is caused by HBV infection and 45% of patients with liver cancer caused by HBV infection [10]. Although many new treatments, such as transcatheter arterial chemoembolization, have been developed in recent years, surgical resection of tumor lesions in recent decades is still the first choice for patients with primary liver cancer. However, the prognosis of patients remains unsatisfactory due to the high rates of postoperative recurrence and metastasis. Determined prognostic biomarkers facilitate the development of individualized treatment strategies for patients. In recent years, with the continuous development of biomedicine and immunopathology, the markers used for diagnosis, disease evaluation, and prognosis have gradually increased. Among them, alpha-fetoprotein (AFP) is a commonly used serum tumor marker, although it has certain specificity. However, there is still a phenomenon of underdiagnosis [11]. Some existing works found that the dynamic changes of immune, nervous, and endocrine systems in patients from HBV infection to tumor formation play an important role [12]. Above achievements lay a theoretical foundation for finding meaningful markers.

Oxidative stress is the state of imbalance between cell oxidation and antioxidation, excessive promotion of oxides, exceeding the scavenging capacity of antioxidants, leading to the accumulation of free radicals in cells and the oxidative damage of biological macromolecules such as proteins, lipids, and DNA, resulting in cell or tissue damage [13]. In previous studies, they found that oxidative stress is involved in the formation of a variety of diseases, such as cancer, diabetes, and cardiovascular and neurological diseases, and in cancer research, others found that oxidative stress may have a high probability of joining in the formation of HCC [14, 15]. Interleukin 6 (IL-6) can inhibit tissue inflammation and cell apoptosis [16], and one of the important functions of tumor necrosis factor *α* (TNF-*α*) is to activate the cell apoptosis pathway. Oxidative stress can induce hepatocyte injury, produce multiple cytokines and chemokines such as IL-6 and TNF-*α*, promote the occurrence of fibrosis, and affect liver inflammation and cell apoptosis [17]. In addition, mitochondrial dysfunction caused by oxidative stress can affect many important functions of hepatocytes, leading to the development of cells towards cancer. Mitochondria are the main endogenous source of ROS in human body. Excessive ROS in human body will directly attack mitochondria. Because mitochondrial DNA (mtDNA) lacks histone protection and complete repair mechanism, mtDNA is sensitive to oxidative stress and vulnerable to ROS interference, resulting in mtDNA mutations, respiratory chain complex degeneration, and oxidative phosphorylation dysfunction. In addition, mitochondrial dysfunction caused by oxidative stress can affect many important functions of hepatocytes, leading to the development of cells towards cancer. A large amount of ROS accumulation would increase the deposition of oxidized lipids, thereby inducing more lipid peroxidation, inhibiting the respiratory electron transport chain, and forming a vicious cycle [18]. The excessive ROS generated in the body attacks the lipid and oxidizes the lipid on the cell membrane surface, resulting in changes in the structure and properties of the cell membrane. MDA is the lipid peroxide formed by ROS attacking the lipid and oxidizing the lipid on the cell membrane surface. Its level can reflect the oxidative stress state of the body. As a natural free radical scavenging system in human body, SOD maintains a dynamic balance with oxygen free radicals under normal conditions and changes with the change of oxygen free radical level and membrane lipid peroxidation under pathological conditions. Uric acid is the product of hydrolysis, deamination, and oxidation of purine nucleotides in human body. Its content is related to the catabolism rate of nucleic acid and excretion function of kidney. Acute kidney injury after advanced liver disease is a common syndrome in clinical practice. Relevant research evidence shows that there is a complex correlation between the liver and kidney [19].

## 3. Object and Method

### 3.1. Source of Research Object

The patients with hepatitis B-related liver cancer treated in our hospital from January 2019 to December 2020 were retrospectively analyzed. The following criteria were included. The pathological diagnosis of liver cancer was confirmed after operation. The patient had a history of hepatitis B and had no other causes of liver cancer such as hepatitis C and alcoholic liver disease. The biochemical indexes of the patient were detected within one week before operation, and the radical resection of liver cancer was performed in our hospital, with complete clinical data and follow-up data. Exclusion requirements combined with the following criteria, patients with severe underlying diseases and other tumors, received other antitumor treatment. All the contents of this study are with the informed consent of patients.

### 3.2. Data Collection and Specific Research Methods

The data collected contain basic information of patients, gender, age, tumor size, tumor number, TNM stage, and BCLC stage. Next, the last blood biochemical examination within a week before surgery, including superoxide dismutase (SOD), malondialdehyde (MDA), and serum uric acid (SUA) are selected as laboratory indicators. The preoperative blood biochemical examination and corresponding clinical pathological data of the patients were collected and included through the hospital case data system. The receiver operating characteristic curve (ROC) was used to analyze and calculate the blood indexes before treatment, followed by the optimal cutoff value for survival prediction. With the cutoff value as the critical value, it was divided into two categories of variables. Single-factor Cox regression model was used to screen the factors affecting the overall survival (OS) of patients and construct the survival curve. The survival differences at different levels of indicators were compared. Finally, multivariate Cox regression analysis was performed.

### 3.3. Follow-Up Method

All cases included in the study were followed up, including outpatient follow-up and telephone follow-up. Liver ultrasound, chest X-ray examination, serum AFP detection, and CT comparison were performed every 6 months after operation [20, 21]. Tumor recurrence and death were recorded within 3 years. Patients who lost follow-up or died for other reasons are defined as deletion. Tumor recurrence is defined by clinical, radiological, or pathological diagnosis [22]. Follow-up continued until death or the deadline for follow-up was December 2021. OS is defined as the time to start treatment to any cause of death [23]. The time of survival or loss of follow-up at the end of follow-up was counted as the final deadline for statistical analysis.

### 3.4. Statistical Methods

The specific steps of statistical methods are as follows.

- Step 1: SPSS 21.0 is applied to analysis data. The collected data that conform to the normal distribution are expressed as mean ± standard deviation. In order to meet the comparison between the standard groups, *t*-test is used.
- Step 2: after K–S test, M(P25, P75) should be adopted to deal with the measurement data that do not conform to the normal distribution. The enumeration data will be replaced, and chi-square (*χ*^2^) test can be used for comparison between groups of those data.
- Step 3: the cutoff values of SOD, MDA, and SUA will be selected as binary variables for Cox regression analysis.
- Step 4: univariate and multivariate Cox regression analysis on the prognostic factors of patients will be performed, and Kaplan-Meier method and log-rank correction test were used. *P* < 0.05 was used as the criterion for statistical difference in the whole study.

## 4. Results and Discussion

### 4.1. Clinical Data of Included Patients

Finally, the study collected 712 patients, including 520 males and 192 females. The age range was 39–73 years old, and the average age was (51.36 ± 8.23) years old. The number of tumors in patients was multiple (≥2), and the average tumor size was (5.12 ± 1.49) cm. The overall survival rates of patients 1 and 3 years after operation were 68.56% and 53.09%, and the total survival time was 2–36 months. The median survival time of patients with large logarithm was 24 months. As of the follow-up date, there were 363 patients with disease recurrence, of which 334 died. There were 323 patients who did not appear the outcome of this study, 26 patients were lost, and the loss rate was 3.65%, as shown in Table 1.

### 4.2. Determination of Optimal Cutoff Values for Preoperative SOD, MDA, and SUA

Referring to the patient's final survival status, the optimal cutoff values of preoperative SOD, MDA, and SUA were 58.055 U/mL, 10.825 nmol/L, and 312.77 nmol/L, respectively. The sensitivity is 0.844, 0.838, and 0.719, respectively. The specificities were 0.778, 0.761, and 0.701, respectively, as shown in Table 2 and Figure 1. According to the preoperative SOD, MDA, and SUA cutoff values, they were divided into high SOD group (≥58.055 U/mL), low SOD level group (<58.055 U/mL), and MDA high level group (≥10.825 nmol/mL), MDA low level group (<10.825 nmol/L), SUA high level group (≥312.77 nmol/L), and SUA low level group (<312.77 nmol/L).

### 4.3. Univariate Analysis of Patient Prognostic Factors

Univariate analysis showed that preoperative TNM stage, SOD < 58.055 U/mL, MAD ≥ 10.825 nmol/L, and SUA ≥ 312.770 mmol/L were the main factors affecting the OS of patients (*P* < 0.05), as shown in Table 3.

### 4.4. Comparison of Survival Curves between Groups

In NM stage group, high and low SOD, MDA group, and high and low SUA group, compared with Log-rank test, we found that the overall survival time was statistically significant among them (*χ*^2^ = 17.213, *χ*^2^ = 26.433, *χ*^2^ = 7.548, *χ*^2^ = 26.683). Figures 2 and 3 show the results of OS comparison by SOD stratification and results of OS comparison by MDA stratification, respectively. In Figure 4, the results of OS comparison in 712 patients with TNM classification can be observed. Besides, Figure 5 demonstrates the results of OS hierarchical comparison by SUA.

### 4.5. Prognostic Factors of 712 Patients Screened by Multivariate Cox Regression Model

Cox multivariate analysis showed that the survival time of patients with SOD < 58.055 U/mL was shorter than that of patients with SOD ≥ 58.055 U/mL, and the survival time of patients with SUA ≥ 312.770 mmol/L was shorter than that of patients with SUA < 312.770 mmol/L. It was confirmed that patients with low levels of SOD and high levels of SOD had worse prognosis. At the same time, TNM staging also had a certain impact on the prognosis of liver cancer. The larger the staging is, the shorter the survival time of patients after operation will be, as shown in Table 4.

## 5. Conclusions

In this study, the ROC curve was used to analyze the optimal truncation values of MDA, SOD, and SUA, which were 10.825 nmol/L, 58.055 U/m, and 312.77 mmol/L, respectively. The patients were analyzed according to different truncation points. From the survival curve, it can be found that the postoperative survival time of patients with MDA < 10.825 nmol/L and SUA < 312.77 mmol/L was higher than that of patients with MDA ≥ 10.825 nmol/L and SUA ≥ 312.77 mmol/L. The overall survival time of patients with SOD ≥ 58.055 U/m was higher than that of patients with SOD < 58.055 U/m. Single-factor results showed that MDA, SOD, SUA, and TNM staging were correlated with prognosis, and Log-rank test results confirmed that the above indicators were correlated with the prognosis of patients. The results of multivariate analysis also showed that preoperative SOD < 58.055 U/mL and SUA ≥ 312.770 mmol/L and TNM staging III-IV were independent risk factors affecting the postoperative prognosis of patients, indicating that the prognosis of these liver cancer patients after radical resection may be poor and the survival time may be shortened.

In general, the preoperative oxidative stress level and serum uric acid are closely related to the death of patients with hepatitis B-related liver cancer after surgical resection. In the future, it is worth paying attention to the preoperative oxidative stress level and serum uric acid in clinical work. Research and detection of SOD and SUA levels in patients before surgery have been carefully evaluated and selected treatment options, which have important clinical significance for judging the prognosis of liver cancer after surgery. It should be noted that more prospective large sample studies are also needed to further explore the optimal predictive thresholds of SOD and SUA for predicting the death of patients and postoperative so as to further improve the predictive efficiency.

## Figures and Tables

**Figure 1:** ROC curve of preoperative SOD, MDA, and SUA as data variables.

**Figure 2:** Results of OS comparison by SOD stratification in 712 patients.

**Figure 3:** Results of OS comparison by MDA stratification in 712 patients.

**Figure 4:** Results of OS comparison in 712 patients with TNM classification.

**Figure 5:** Results of OS hierarchical comparison by SUA in 712 patients.

**Table 1:** Clinical data of 712 patients.

Factors	$\left(\bar{\chi }\pm s\right)$ /*n*(%)/M(P25, P75)
Sexuality	
Males	520 (73.03)
Female	192 (26.97)
Age (years old)	51.36 ± 8.23
Tumor size (cm)	5.12 ± 1.49
Number of tumors	
1	164 (23.03)
≥2	548 (76.97)
TNM staging	
I ∼ II	413 (58.01)
III ∼ IV	299 (41.99)
BCLC staging	
0 ∼ A	85 (11.94)
B	313 (75.97)
C	314 (12.09)
SOD (U/mL)	60.12 ± 14.36
MDA (nmol/L)	8.89 ± 1.02
SUA (mmol/L)	312.45 ± 89.36
OS (month)	24 (11, 36)

**Table 2:** ROC curve parameters of preoperative SOD, MDA, and SUA prompting the prognosis of patients.

Factors	AUC	Sensitivity	Specificity	Youden index	Cut-off	*P* value
SOD	0.844	0.851	0.778	0.629	58.055	<0.001
MDA	0.838	0.842	0.761	0.603	10.825	<0.001
SUA	0.719	0.683	0.701	0.390	312.770	<0.001

**Table 3:** Univariate analysis of overall survival of patients.

Factor	HR	95% CI	*P* value
Sexuality			
Male	1		
Female	1.094	0.816, 1.467	0.548
Age (years old)			
<51	1		
≥51	1.033	0.770, 1.387	0.828
Tumor size(cm)			
<5	1		
≥5	1.494	1.110, 2.013	0.066
Number of tumors			
1	1		
≥2	1.715	1.011, 2.654	0.062
TNM staging			
I ∼ II	1		
III ∼ IV	1.830	1.109, 3.020	0.018
BCLC staging			
0 ∼ A	1		
B	1.997	0.432, 9.242	0.376
C			
SOD (U/mL)			
<58.055	1		
≥58.055	4.471	2.217, 9.017	<0.001
MDA (nmol/L)			
<10.825	1		
≥10.825	1.704	1.014, 2.863	0.044
SUA (mmol/L)			
＜312.770	1		
≥312.770	1.874	1.108, 3.170	0.019

**Table 4:** Prognostic factors of 712 patients screened by multivariate Cox regression model.

Factor	HR	95% CI	*P* value
TNM staging (I ∼ II are controls)	1.555	1.172, 2.063	0.002
SOD (<58.055 U/mL are controls)	1.533	1.154, 2.036	0.003
MDA (<10.825 nmol/L are controls)	1.300	0.978, 1.728	0.071
SUA (<312.770 mmol/L are controls)	1.612	1.215, 2.138	0.001

## Data Availability

The data used in the paper are available from the corresponding author upon request due to requirements of permission and consent.

## References

[1] Qiu W. Q., Shi J. F., Guo L. W. (2018). Medical expenditure for liver cancer in urban China: a 10-year multicenter retrospective survey (2002-2011). *Journal of Cancer Research and Therapeutics*.

[2] Akateh C., Black S. M., Conteh L. (2019). Neoadjuvant and adjuvant treatment strategies for hepatocellular carcinoma. *World Journal of Gastroenterology*.

[3] Chong C. C. N., Wong G. L., Lai P. B. (2014). Impact of antiviral therapy on post-hepatectomy outcome for hepatitis B-related hepatocellular carcinoma. *World Journal of Gastroenterology*.

[4] Sharma A., Rajappa M., Saxena A., Sharma M. (2007). Antioxidant status in advanced cervical cancer patients undergoing neoadjuvant chemoradiation. *British Journal of Biomedical Science*.

[5] Trindade D. B., de Araújo V. A., Franco E. P., Fernandes R. C., Carvalho A. P. P. F., Pimentel G. D. (2020). Serum uric acid concentration is not associated with handgrip strength, lean body mass or survival in gastrointestinal cancer patients. *Clinical Nutrition ESPEN*.

[6] Chong F., Huang J. J., Huang N. N. (2020). Associations between serum uric acid and hepatobiliary-pancreatic cancer: a cohort study. *World Journal of Gastroenterology*.

[7] Yadav K. D., Patil B. A., Raheel S. A. (2020). Serum uric acid levels in patients with oral cancer, leukoplakia and submucous fibrosis: a cross-sectional study. *Translational Cancer Research*.

[8] Jiang M., Ren L., Chen S., Li G (2021). Serum uric acid levels and risk of eight site-specific cancers: a mendelian randomization study. *Frontiers in Genetics*.

[9] Lombardi R., Pisano G., Fargion S. (2016). Role of serum uric acid and ferritin in the development and progression of NAFLD. *International Journal of Molecular Sciences*.

[10] Wang F. S., Fan J. G., Zhang Z., Gao B., Wang H. Y. (2014). The global burden of liver disease: the major impact of China. *Hepatology*.

[11] Luo P., Wu S., Yu Y. (2020). Current status and perspective biomarkers in AFP negative HCC: towards screening for and diagnosing hepatocellular carcinoma at an earlier stage. *Pathology and Oncology Research*.

[12] D’souza S., Lau K. C., Coffin C. S., Patel T. R. (2020). Molecular mechanisms of viral hepatitis induced hepatocellular carcinoma. *World Journal of Gastroenterology*.

[13] Saha S. K., Lee S. B., Won J. (2017). Correlation between oxidative stress, nutrition, and cancer initiation. *International Journal of Molecular Sciences*.

[14] Lee J., Giordano S., Zhang J. (2012). Autophagy, mitochondria and oxidative stress: cross-talk and redox signalling. *Biochemical Journal*.

[15] Wang Z., Li Z., Ye Y., Xie L., Li W. (2016). Oxidative stress and liver cancer: etiology and therapeutic targets. *Oxidative Medicine and Cellular Longevity*.

[16] Yu H., Pardoll D., Jove R. (2009). STATs in cancer inflammation and immunity: a leading role for STAT3. *Nature Reviews Cancer*.

[17] Djordjevic J., Djordjevic A., Adzic M., Niciforovic A., Radojcic M. (2010). Chronic stress differentially affects antioxidant enzymes and modifies the acute stress response in liver of Wistar rats. *Physiological Research*.

[18] Ahmad S. T., Arjumand W., Nafees S. (2012). Hesperidin alleviates acetaminophen induced toxicity in Wistar rats by abrogation of oxidative stress, apoptosis and inflammation. *Toxicology Letters*.

[19] Chancharoenthana W., Leelahavanichkul A. (2019). Acute kidney injury spectrum in patients with chronic liver disease: where do we stand?. *World Journal of Gastroenterology*.

[20] DeBerardinis R. J., Chandel N. S. (2016). Fundamentals of cancer metabolism. *Science Advances*.

[21] Yu T. Y., Jin S.-M., Jee J. H., Bae J. C., Lee M.-K., Kim J. H. (2019). The protective effects of increasing serum uric acid level on development of metabolic syndrome. *Diabetes & Metabolism Journal*.

[22] Wang H., Zhang H., Sun L., Guo W. (2018). Roles of hyperuricemia in metabolic syndrome and cardiac-kidney-vascular system diseases. *American Journal of Tourism Research*.

[23] Oral A., Sahin T., Turker F., Kocak E. (2015). Relationship between serum uric acid levels and nonalcoholic fatty liver disease in non-obese patients. *Medicina (Rijeka)*.

